# Tamarind: A diet‐based strategy against lifestyle maladies

**DOI:** 10.1002/fsn3.1218

**Published:** 2019-09-27

**Authors:** Muhammad Sajid Arshad, Muhammad Imran, Aftab Ahmed, Muhammad Sohaib, Azmat Ullah, Mehr un Nisa, Gule Hina, Waseem Khalid, Hafiza Rehana

**Affiliations:** ^1^ Institute of Home and Food Sciences Government College University Faisalabad Pakistan; ^2^ Department of Diet and Nutritional Sciences University of Lahore Lahore Pakistan; ^3^ Department of Food Science and Human Nutrition University of Veterinary and animal Sciences Lahore Pakistan

**Keywords:** anticancer, antioxidant status, health perspectives, tamarind, tamarind kernel powder

## Abstract

The modern‐day review article is an exquisite attempt to demonstrate the extreme therapeutic potential of tamarind fruit (*Tamarindus* *indica*), particularly its pulp, seed, and leaf extract, against lifestyle‐related chronic disorders. The rapid transition in the diet patterns and also the varying lifestyle of the people has made its way forth, a momentous upsurge in a number of chronic as well as degenerative diseases. An excess of foods having functional and nutraceutical significance has come into view recently. These foods have emerged as effective therapeutical remedies against these disorders owing to their natural phytochemical constituents present in them, in abundance. *Tamarindus* *indica* serves as a proverbial herbal medicine in each and every part of the world that is known to mankind. Also, the tamarind kernel powder (TKP) is of immense commercial significance in some of the major, leading industries of the World. The derivation of an important gel‐forming substance (polysaccharide), named as “jellose,” from the decorticated seed kernels of tamarind fruit has led to the manufacture of pectin. It is used in industrial scale in the preparation of various products like jams, jellies, and most important in the preparation of cheese. It plays an evident role as a stabilizer of commercial significance, and it has also been greatly recommend by the scientists to be used as a potent ingredient in a range of pharmaceutical products. The leaves of tamarind plant are also used as part of the daily diet in several countries where they are readily consumed in fresh form and especially during drought season.

## 1 INTRODUCTION

*Tamarindus* *indica* (*T. indica*) that is commonly known as tamarind belongs to the dicotyledonous “Leguminosae” Family (Lewis, Schrire, Mackinder, & Lock, 2005) and for obtaining pulp from its fruit, which is used for the preparation of a beverage and to add flavor to curries, sauces, and confections, its cultivation is chiefly done. T. indica is a proverbial herbal medicine in almost every part of the world known to mankind (Siddhuraju, 2007). The pulp obtained from tamarind fruit is mostly consumed fresh and is made into juice, brine, or infusion as well, and it is also used in the preparation jams and sweets; it can also be processed. The tamarind kernel powder (TKP), the most important and useful sizing material which is used in some of the prominent industries like the paper‐making industry, textile, and jute industry also, is therefore regarded as the key product of tamarind seed having industrial significance (Kumar & Bhattacharya, 2008). The principal raw material used in the manufacture of the polysaccharide “jellose,” tannin and adhesive also, comes from the tamarind seed. It was revealed by the two Indian Scientists in 1942 that there was the presence of a gel‐forming substance in percentage of 46–48, in the decorticated seed kernels of tamarind fruit. As named “jellose,” this polysaccharide (pectin) is now being employed as a stabilizer in the commercial production of cheese, ice cream, and mayonnaise because of its jelly (gel)‐forming properties and carbohydrate nature (El‐Siddig et al., 2006), plus it has also been recommended by scientists to be used as an agent or as a potential ingredient in the manufacture of various pharmaceutical products. Cakes and breads are also made by using the flour that is obtained by the seed of tamarind. As far as the flavor is concerned as compared to groundnuts, the seeds of tamarind which are roasted and then used are stated to be as more superior (ICRAF, 2007). The leaves and flower of tamarind are being consumed as fresh, raw vegetables by people in many regions and can also be made into a variety of restaurant quality dishes (ICRAF, 2007). They are also used to make salad dressings, soups, stews, and curries in many countries such as India, Nigeria, Nepal, Bangladesh, and Sudan, particularly during drought and dearth times (El‐Siddig et al., 2006).

The plant of tamarind is being employed as a worthy conventional (traditional) medicine in many tropical countries but most significantly in countries such as Bangladesh, India, Sudan, and Nigeria (Ferrara, 2005; Kristensen & Balslev, 2003) T. indica contains crude protein in extremely high amount/levels. As it holds an elevated level of proteins in conjunction with several other essential amino acids, it is because of this reason that these contribute a great deal in building strong and capable muscles. *Tamarindus* *indica* is also rich in energy‐providing carbohydrates and also in some minerals, just like calcium, potassium, phosphorus, and magnesium in high amounts. It can provide vitamin A and iron in smaller amounts as well. As whole of the tamarind plant is used expansively for many industrial and medicinal purposes, therefore, it is considered extremely beneficial for the health of human beings (Yanez, Zacarias, Aguayo, Vasquez, & Guzman, 1995). The presence of a large number of many active constituents was uncovered as a consequence of the phytochemical investigation that was carried out on T. indica plant. These constituents included phenolic compounds, uronic acid, L‐(‐)malic acid, tartaric acid, pectin and mucilage, cardiac glycosides the mucilage, plus arabinose, xylose, glucose, and galactose. The incidence of a variety of such elements which are essential like calcium, copper, iron, cadmium, manganese, arsenic, sodium, magnesium, potassium, phosphorus, zinc, and lead and also fatty acids was shown by the ethanolic extract of *T. indica* (Coutino‐Rodriguez, Hernandez‐Cruz, & Gillis‐Rios, 2001). The pulp of tamarind fruit contains some of the crucial organic acids which include tartaric acid most importantly, plus citric acid and acetic acid, malic acid, succinic acid as well as formic acid, also amino acids, invert sugar in the percentage of 25%–30%; proteins, pectin, and fat; a few pyraines (trans‐2‐hexenal), as fragrant some thiazoles which include 2‐ethylthiazole and 2‐methylthiazole; moreover, with a main chain consisting of β‐1,4‐connected glucose molecules in conjunction with xylose (alpha‐1,6) and galactose; total protein; lipids with fatty oils; and some keto acids, the seed polysaccharides are formed. In addition to this, lupanone and lupeol, the two triterpenes were also present in the leaves of the plant (Imam, Azhar, & Hasan, 2007; Samina et al., 2008).

The tamarind pulp industry gives off tamarind seed, in the form of its by‐product. In recent times, the tamarind industry discarded surplus amount of tamarind seed waste (Oluseyi & Temitayo, 2015). Tamarind seed itself is immensely rich in phytochemicals which comprise of phenolic antioxidants, for example, catechin, epicatechin, 2‐hydroxy‐3′,4′‐dihydoxyacetophenone,3,4‐methyl‐dihydroxybenzoateand 3,4‐dihydroxyphenyl acetate. The antioxidant potential is also being exhibited the TSE’s via plummeting the peroxidation of lipids (in vitro) and the antimicrobial activity. Consequently, the seed of tamarind has the potential of providing nutritional and nutraceutical value comprising of low cost (Andabati & Muyonga, 2014).

The investigation for phytochemicals done on the root bark of *T. indica* showed the incidence of (+)‐pinitol, eicosanoic acid, *n*‐hexacosane, b‐sitosterol, octacosanyl ferulate, and 21‐oxobehenic acid. For the very first time, the presence of the bioactive compound known as (+)‐pinitol, in tamarind plant, is being reported (Jain, Jain, Sharma, Hideyuki, & Hatano, 2007; Pino, Escalora, & Licea, 2002). The fruit pulp volatile constituents, that is, (44.4%) and (33.3%) of the total volatiles, were furan and carboxylic acid derivatives, respectively (Warda, Fathia, & Amel, 2007). The majority of the fatty acids present in the seeds of tamarind fruit were oleic, linoleic, palmitic, and eicosanoic acids. The incidence of β‐amyrin, β‐sitosterol, campesterol, plus seven significant hydrocarbons was shown by the residual unsaponifiable matter obtained through T. indica seed oil. The presence of acids which include acetic acid, succinic acid, and tartaric acid plus sugar, gums and pectin, tannins, alkaloids, flavonoids, glycosides, and sesquiterpenes was demonstrated by the Aerial parts of this plant (Aida, Rosa, Blamea, Thomas, & Salvador, 2001). The polyphenolic profile in the pericarp of tamarind leaves in several different forms just like apigenin, catechin, epicatechin, procyanidin B2, procyanidin dimer, and trimer, together with naringenin, eriodictyol, and taxifolin of total phenols, respectively, was dominated by the proanthocyanidins. The tamarind seed content consisted of procyanidins only, primarily represented by the “oligomeric” procyanidin tetramer, procyanidin hexamer, and procyanidin pentamer with B2 epicatechin procyanidin, present in small amounts (Sudjaroen et al., 2005). The pericarp and seed of tamarind plant contained polyphenolic compounds. The total yield of polyphenolic compounds in seeds was 6.54 g/kg, by using the Soxhlet extraction with CH_3_OH (methanol), and in pericarp, it was found to be about 2.82 g/kg. The pericarp contained polyphenolic compounds which were present in the following forms, that is, procyanidin B2 being 8.1%, catechin being 1%, epicatechin being 9.2%, and procyanidin trimmers up till procyanidin‐hexamers and apigenin, eriodyctyol, naringenin, luteolin, and taxifolin like flavonoids were dominated by proanthocyanidins (73.4%) (Kuru, 2014; Sudjaroen et al., 2005; Yamin, Sobiya, Fayyaz, & Muhammad, 2011).

## 2 ANTIOXIDANT STATUS

Antioxidants are of much use in providing protection against the damage caused by oxidation. They are really important in preventing the build‐up of the free radicals and as a consequence oxidative damage in the human body. Plants are the rich alternative sources of the naturally occurring antioxidants, and they can therefore complement the antioxidants that are produced by the human body itself (Razali, Mat Jonit, Ariffin, Ramli, & Abdul, 2015). Principally, due to its free radical scavenging activity and also the protection that is provided in opposition to the induced stress as a result of oxidation process (oxidative stress), the antioxidant activity in this way plays a very important part in the sustenance of human health (Haghju & Almasi, 2015; Valdes et al., 2015). By the presence of this antioxidant activity, the development of diseases, which include coronary heart diseases, are readily prevented (Farias, Guzmán‐Martínez, Delgado, & Maccioni, 2014; González‐Vallinas, González‐Castejón, RodríguezCasado, & Molina, 2013).

The pulp of tamarind is rich in numerous phytonutrients that serve as potent dietary antioxidants; these phytonutrients together with the total phenolic content showed a very strong correlation (Khairunnuur et al., 2009). In contrast to the avocado, jackfruit, mango, and longan fruit flesh, the tamarind flesh showed greater phenolic content as demonstrated by Soong and Barlow in 2004. The fruit extract of tamarind enhances the efficacy of antioxidant defense system present in the body. Therefore, in humans, this extract has now gained the potential to control and limit the risk of atherosclerosis development (Martinello et al., 2006). This fruit extract can also be frequently used in the treatment of abdominal pain and as a laxative (Havinga et al., 2012). Because of its properties which include lower expenditures of logistics, easy to use form and longer shelf life due to low water activity (Aw), the tamarind powder has thus become a product of great interest (Jittanit, Chantara, Deying, & Ratanavong, 2011).

Also, the crude (raw) extract of tamarind pulp contains phenolic compounds. These phenolic compounds obtained from the pulp extract, when administered to animals, largely improved the effectiveness of certain enzymes for instance glutathione peroxidase, superoxide dismutase, and catalase, due to the strong antioxidative properties associated with them (Lim, Junit, Abdulla, & Aziz, 2013; Martinello et al., 2006). In the seed coat's ethanolic extract, which is a by‐product of the tamarind gum industry, there is also presence of antioxidant activity and this extract can be used as a valuable source of many inexpensive and safe antioxidants (Razali et al., 2015). The leaves of *Tamarindus* *indica* (plant) are rich in fatty acids, lipids, flavonoids, and vitamins as well. These leaves of tamarind plant have an enormous potential as effective medicinal products’ source, primarily due to this high number of beneficial components that they contain, still with the existence of such compounds like saponins, which are recognized largely on behalf of the presence of their metabolites, which can powerfully initiate the cell breakdown. Escalona (Escalona‐Arranz et al., 2010) alternatively examined the pharmacological properties of the extract plus the toxicity caused by the tamarind leaves extract in erythrocytes. Thus, the results depicted that possibly due to their antioxidative mechanisms and rich flavonoid amount, no harmful properties were observed even with the incidence of saponins; in addition, they detected that the extract worked effectively and turned out to be source of the protection of cells from lysis (Gunaseelan, 2016). The investigation carried out by Razali et al. (2015) acknowledged the existence of several polyphenolic components in the extract of seed. With respect to the antioxidant activity, they found caffeic acid as the most active compound that has been identified in aging process and in many other common diseases nowadays, which include diabetes, inflammatory diseases, cardiovascular diseases (CVD’s), and cancer therefore able to protect cells against lipid peroxidation. According to another research, the coat of T. indica seed contains some of the dynamic antioxidants, like flavonoids, phenolics, and tannins, and some beneficial activities such as lipid peroxidation reduction, collagen‐stimulating antityrosinase, antidiabetic, antimicrobial, anti‐inflammatory, and antihyperlipidemic activities are also being possessed by its extracts.

Sundaram et al. (2015) showed that, by the bone degeneration mediators, inflammation of cartilage and oxidative stress regulation, the seed extract improved arthritis. The disparity (Arthritis) is associated with the degradation by enzymes of subchondral bone and the important articular cartilage by means of matrix metalloproteinases abbreviated as MMP’s, exoglycosidases and hyaluronidases. The upsurge in the activity of these enzymes is inhibited by the use of the tamarind seed extract. The seeds of tamarind also possess a natural polysaccharide known as xyloglucan, which is used in some important industries like food and the pharmaceutical (medicine) industry (Hirun, Sangfai, & Tantishaiyakul, 2015).

## 3 HEALTH PERSPECTIVES OF TAMARIND

### 3.1 Anticancer

The Renal Cell Carcinoma, commonly called as RCC, is one of the most widely spread malignancies of the adult kidney. RCC lacks early signs and therefore at the first stage of diagnosis, often results in metastasis. A compound N di‐ethyl nitrosamine also called DEN instigated and another component ferric nitrilotriacetate also termed as FeNTA‐stimulated RCC can possibly act as a convenient, useful, and efficient experimental model; however, this model is not fully characterized. All through the RCC development, at different times the alterations in histology and markers of oxidative stress were completely analyzed, through this study, in the light of current classification, the histological subtype was re‐evaluated and the effect of seed extract of tamarind (TSE) was observed. The investigational groups of the Wistar rats (male) were DEN + FeNTA, TSE + DEN+FeNTA, TSE, and DEN. Two weeks before the administration of DEN (200 mg/kg) and all through the experiment, TSE was given to these groups. The two FeNTA doses of 9 mg Fe per kg for nephrotoxicity (acute) and enhancing FeNTA doses 3 to 9 mg Fe per kg two times in a week, approximately for a period of 16 weeks for carcinogenesis protocol, after fourteen days of DEN treatment were being administered. Necrosis and renal failure were observed in the acute study and the use of tamarind seed extract (TSE) ameliorated these conditions. Ever since 1 month of FeNTA treatment, the preneoplastic lesions were observed, during the carcinogenesis protocol at the second month, were even more obvious when the renal cysts and RCC were already detected as well. The RCC tumors were attained with no evident variations in kidney function; in addition, a clear histological cell subtype was recognized in all the cases. The compound 4‐hydroxy‐2‐nonenal as well as 3‐nitro‐L‐tyrosine intensities amplified progressively during the procedure. Tamarind seed extract reduced both the oxidative stress markers, and it also delayed the progress of RCC and decreased its incidence by (21%) although there was no statistical difference (Sanyasi, Kumar, Goswami, Bandyopadhyay, & Goswami, 2014; Vargas‐Olvera et al., 2012).

The antitumor action of the PST001a polysaccharide sequestered from *Tamarindus* *indica* seed kernel was observed. The various cell lines for cancer like A549, MCF‐7, and KB of humans as well as DLA and EAC similar cell lines of murine were cured with the extracted component (PST001), and by using the MTT assay, amelioration of cell growth was gauged. Several in vivo investigations were performed for assessing harmfulness, immunemodulation, and tumor retardation or cessation. The results revealed that respective IC (50) of component in A549, DLA, and KB was at 80.62, 91.13, and 190 (μg/ml). In both tumors, that is, DLA and EAC, on treatment with the polysaccharide PST001, significant reduction in the tumor was obtained, and this reduction was even further protuberant when this polysaccharide was directed along with the compound 5‐fluorouracil. The results depicted that surge in WBC and T‐cell population (CD 4+), and for this compound, the bone marrow cellularity consequently evoked robust immunomodulatory activity. The toxicological studies did not reveal the presence of any major abnormality (Aravind, Joseph, Varghese, Balaram, & Sreelekha, 2012; Choy et al., 2016; Shilpi et al., 2015; Shivshankar & Shyamala Devi, 2004).

In humans, the administration of procyanidin (10–40 μM) in prostate microvascular endothelial cells (HPMECs) and endothelial cells of umbilical vein (HUVECs) retards growth and causes the stimulation of death in both types of these cells, that is, HUVECs and HPMECs. It was discovered by additional studies that by the downregulation of CDKs (Cdk2, Cdc2), Cdc25c phosphatase, and D1 plus A cyclins, and by the upregulation of the CDK inhibitors (p21, p27) expression, a G1 arrest in the cell cycle progression of HUVECs was caused by B2G2.Via, increasing the p53, Smac/Diabl and Bax expression and through decreasing the surviving and Bcl‐2 levels, B2G2 induced strong apoptotic death in HUVECs. In addition to this, in HUVECs and HPMECs, the capillary tube formation induced by growth factors was also inhibited by B2G2. Interestingly, the conditioned media as grown under normoxic (**~**21% O_2_) and hypoxic (1% O_2_) conditions, from the prostate cancer (PCA) cells PC3 and LNCaP, significantly enhanced the capillary tube formation in HUVECs, which in the presence of conditioned media from the B2G2‐treated PCA cells was being compromised. The invasiveness and the motility of both cells, the HUVECs as well as HPMECs, were also inhibited by B2G2 (Kumar, Deep, Wempe, Agarwal, & Agarwal, 2015).

In the esophageal adenocarcinoma (OA) cells, the JNK and p38 activation together with the expression and phosphorylation of c‐Jun were induced by procyanidin. The inhibition of the activity of JNK but not that of p38 kinase activity thus prevented the expression and phosphorylation of c‐Jun was induced by procyanidin. Also, the effects induced by procyanidin on apoptosis and cell proliferation were diminished by the knockdown of the JNK1, JNK2, or JUN gene expression. The “c‐Jun” is a constituent of the transcription factor AP‐1, and the AP‐1 binding sites in the promoters of genes that were induced by procyanidin are over presented. This indicates that in OA cells the induction of apoptosis is brought about by the JNK activation of c‐Jun, by procyanidin, and it also suggests a role for the transcriptional program mediated by c‐Jun (Connor, Adriaens, Pierini, Johnson, & Belshaw, 2014). Luteolin demonstrated strong anticancer activity via reduced breast cancer cell metastasis, on MDAMB231 human breast cancer cell line (Naso et al., 2016). Likewise, in JEG‐**3** as well as JAR cells, the loss of the mitochondrial membrane potential and apoptosis was induced by luteolin in such a manner which is dependent on the dose. By the treatment of the JAR and JEG‐3 cells with luteolin in such a manner which is dependent on dose and time, the PI3K/AKT pathway was also inhibited. Next, within the existence of the mTOR, ERK1/2MAPK, and P13K/AKT pharmacological inhibitors, we established luteolin effects on the JEG‐3 and JAR cell proliferation. By establishing the effects of luteolin, the expression of mRNA SREBP1 and SREBP2 was considerably reduced; however, only the SREBP1 protein was considerably influenced. Consequently, in the treatment of choriocarcinoma cells present in humans, luteolin plays a vital role by collectively inhibiting the cascade of PI3K, AKT, mTOR, SREBP (1 and 2), and the expression of lipogenic genes (Lim et al., 2013).

The induction of cell apoptosis and inhibition of cell migration by luteolin revealed its remarkable anticancer effects particularly against lung cancer whether the activated protein kinases by mitogen which is abbreviated as MAPKs as well as signaling pathways of Akt are essentially required. The findings thus demonstrated that the compound luteolin in A549 lung adenocarcinoma cells exerted and proliferation protective effect in a dose as well as time‐related manner caused occurrence of apoptosis with a related increase in the activation of caspases (9 and 3), Bcl‐2 dimunition, Bax expression elevation, MEK phosphorylation along with its downstream kinase namely ERK and the activation of Akt. Luteolin also substantially repressed the migration and motility in A549 cell (Meng, González‐Abuín, Pinent, Ardévol, & Blay, 2016).

The benzo(a)pyrene 50 mg/kg body weight given to mice caused elevation in lipid peroxide levels, markers of specific tumor to lungs such as carcinoembryonic antigen also called CEA and NSE or neuron‐specific enolase with an associated decrement both enzymatic antioxidants including superoxide dismutase, glutathione reductase catalase, glutathione‐s‐transferase, glutathione peroxidase, and nonenzymatic antioxidants, for example, reduced glutathione, vitamin C, and vitamin E. Luteolin treatment at 15 mg/kg body weight orally significantly offsets all these harmful alterations and thus maintained normalcy in cells. Besides, the treatment with luteolin was proposed to effectively negate benzo‐a‐pyrene‐induced enhanced regulation of the proliferating cell nuclear antigen expression, nuclear factor‐kappa B (NF‐κB), and cytochrome P450 1A1 was exposed by the evaluation of protein expression by Western bolt method (Han et al., 2016; Kasala, Bodduluru, Barua, & Gogoi, 2016; Yan, Wei, Song, Jia, & Zhang, 2016)).

### 3.2 Antimicrobial role

Many food products during their manufacture, storage, packaging, and distribution often need protection from spoilage by microbes and deterioration because of their perishable nature, to give them the desired shelf life. The preservation of food is an incessant and constant fight against the food spoiling microorganisms or those organisms that make the food unsafe for use and consumption. The most common and frequently used, traditional preservative agents include weak organic acids, like lactic acid, benzoic acid, sorbic acid, and acetic acid. Because of their residues that transpire in the food, these chemical preservatives can therefore prove to be harmful to health. An increasing number of consumers have a preference for the minimally processed foods, prepared with no added chemical preservatives. A totally transformed and improved awareness and interest in the “natural preservation” of food and food products comes out to be stimulated by the present food safety concerns, rise in the production of minimally processed foods coupled with the “green” image policies of the food industries as well as the growing problems with increased resistance of microbes (Chen, Deng, & Li, 2013). The aqueous‐ethanolic extracts of tamarind are effective against *Staphylococcus* *aureus*, *Staphylococcus* *epidermidis*, *Bacillus* *subtilis,* and *Listeria* *monocytogenes*, with an inhibition zone of 18, 19, 16, and 16 mm, respectively, because of the presence of tannins, terpenoids, and citric acid. It also not only inhibited all Gram‐negative bacteria isolate growth but in the case of *Pseudomonas* *aeruginosa*, Pseudomonas sp. and Salmonella sp. produced an inhibition zone greater than 15 mm (Gupta, Prakash, & Gupta, 2014). The minimum inhibitory concentration (MIC) (50, 100, 250, and 500 mg/ml) of the extract of tamarind was used for the observance of antibacterial activity against the test organisms. The highest zone diameter of inhibition given by the methanol fruit extract was 41 ± 1.0 mm for *E. coli* and 37 ± 0.4 mm for *S. typhi* at 500 mg/ml, while the methanol leaf extract gave 0.0 mm for *E. coli* and 25 ± 0.4 mm for *S. typhi* at 500 mg/ml. The methanol and aqueous fruit extracts were effective against the species of *E. coli*, *S. typhi*, and *P. aeruginosa*. The extract of ethanol was effective against *E. coli*, *S. typhi*, *P. aeruginosa*, and *S. aureus*. The ethanolic and methanolic leaf extracts were both effective against *S. typhi* and *P. aeruginosa* species (Ugoh & Jaruma, 2013). The pulp polyphenols of *T. indica *have been proven effective against *B. subtilis* and other human pathogenic microorganism (Anu & Banerjee, 2014).

The seeds of tamarind were used and meant for the ocular delivery of rufloxacin (0.3%) in the treatment of experimental *P. aeruginosa* and *S. aureus* keratitis, in rabbits. The intra‐aqueous penetration of rufloxacin was significantly increased using polysaccharide in both infected and uninfected eyes. The number of *P. aeruginosa* and *S. aureus* in the cornea of the eye lessened at a higher rate via rufloxacin delivered by the polysaccharide than that obtained by simply using rufloxacin. Above all, even when the time interval between different administrations of the drug was extended, the use of polysaccharide allowed a substantial reduction of *S. aureus* species in the cornea to be achieved. These results propose that the polysaccharide of the *T. indica* seed prolongs the precorneal residence times of antibiotics and also enhances the accumulation of drug in the cornea, possibly by reducing the topically administered drugs’ washout. The seed polysaccharide of T. indica appears to be a potential promising candidate, as a vehicle for the topical treatment of bacterial keratitis (Ghelardi, 2004). The ethanolic extract that was hot and aqueous extract that was cold of fruit pulp, stem bark, and leaves of tamarind are of efficient use against the species of *B. subtilis* ATCC, *P. aeruginosa*, *E. coli*, and *B. subtilis* (Nwodo, Obiiyeke, Chigor, & Okoh, 2011).

The alcoholic extract of *T. indica *seeds (200 µg/ml) exhibited the antibacterial activity against *P. aerugnosia*, *E.* *coli*, *S. dysentery*, *S. typhi*, Enteriococcus sp., *S. auerus*, and *B. subtilu*s. The species *S. typhi* and *E. coli* were more susceptible to the seed extract when compared to other bacterial isolates with the inhibition zone up to 35 mm. The presence of alkaloid, flavonoid, saponins, glycosides, and terpenoids was revealed by the phytochemical analysis, while the absence of tannins was found in the extract of seeds. It was indicated by the results that all the bacterial isolates at different degrees have the ability to adhere to smooth surface (plastic and glass tubes). This ability of all the bacterial isolates to stick on and remain in the tubes that are made of glass or plastic was shown to be significantly higher in the case of glass tubes (glass surface) than in plastic tubes (polystyrene surface). Apart from other bacterial isolates, high adherent growth was shown by *E. coli*, *P. aerugnosia*, *S. typhi,* and Enteriococcus species. Furthermore, reduction in the adherent growth of the tested bacteria caused by the seed extract (100, 200 µg/ml) was also found. These results revealed that the ability to form biofilm with diverse degree of thickness and absorbance value range (1.7–0.8) is being possessed by all the tested bacteria. *S. typhi*, *P. aerugnosia*, and *Enteriococcus* showed high production of biofilm with the absorbance values as 1.7, 1.25, and 1.08, respectively (Fouad Rasheed, 2014). The L. leaf extracts of *T. indica* made with 30% as well as 70% ethanol and water, and pure potent essential oil obtained as a result were readily effective against *E. faecalis*, *S. aureus*, *B. subtilis*, *E.coli*, *S. typhirium*, *C. albicans,* and *P. aeruginosa*. The fluid extracts were formerly categorized in a different way for the determination of their total phenolic and flavonoid contents by spectrophotometer, whereas by using gas chromatography/mass spectroscopy (GC/MS), the essential oil was evaluated chemically (Escalona‐Arranz et al., 2010).

### 3.3 2‐Oxidative stress

The tamarind seed coat extract known commonly as “TSCE” imparts effects on the normal skin fibroblast CCD‐1064Sk cells of the humans, by attenuating the intracellular reactive oxygen species (ROS) and enhancing the levels of glutathione (GSH), antioxidative enzymes such as glutathione peroxidase (GPx), superoxide dismutase (SOD), plus the catalase activity (Nakchat, Chai, Li, Zhu, & Huang, 2014).

Tamarind seed extract (TSE) rich in procyanidin prevented the activation of T and B cells in the liver, macrophages, and the inflammatory mediators such as TNF‐α, IL‐1β, and IL‐6 aggravates. It significantly inhibits the burst of oxidation in the liver and helps in maintaining homeostasis (Sundaram et al., 2015). The administration of the leaf powder (2.5, 5, and 10 g %) of *T. indica* caused notable improvements in the lipid and carbohydrate profiles when used for a duration of 4 weeks, as evidenced by the decrease in lipid and plasma glucose levels, lipid peroxidation levels, hexokinase enzyme activity, and excretion of cholesterol and increased hepatic glycogen level, together with simultaneous improvement in both renal and hepatic tissues antioxidant profiles (Vasant & Narasimhacharya, 2012). In the same way, administration of the decoctions made with the leaves of *Tamarindus* *indica* (TI) in the amount 25, 50, and 100 mg/kg, for a period of approximately seven days against acute ethanol (EtOH)‐induced injury of liver, alleviated the activation of EtOH‐induced liver caspase‐3 (42%, 57%, and 64%) as well as fragmentation of DNA (32%, 47%, and 50%), respectively (Ghoneim & Eldahshan, 2012). *Tamarindus indica* along with antioxidant effect also possess the blood glucose‐lowering effect and protective effect on renal complications that are associated with hyperglycemia (Aengwanich & Suttajit, 2010; Agnihotri & Singh, 2013).

The fruit pulp extract of tamarind inhibited the activity of the NADPH oxidase of neutrophils that was assessed by the depletion of O_2_, elastase activity, and degranulation was assessed by different spectrophotometric methods at applications of higher than 200 micrograms per 10 cells (Paula et al., 2009). In the HepG2 cells present in liver, the tamarind polyphenols regulated the expression ofALDH6A1, KNG1, SERPINC1, SERPIND1, SERPINE, FGA, FGG, DHCR24, MVK, CYP24A1, EPHX1, and LEAP2. Moreover, the proteins were involved in the intrinsic prothrombin activation pathway (KNG1, SERPINE1, and FGG), immunoprotection or response (IFNGR1, MX1, LEAP2, and ANXA3) and super pathway of cholesterol biosynthesis (MVK), the xenobiotic metabolism signaling (ALDH6A1, ADH6), and the coagulation system also, and their expression was also altered by it. Conclusively, the leaf extract of tamarind which is rich in antioxidants inhibited the lipid peroxidation and the ROS production, augmented the antioxidants activities related to enzymes, and drastically up surged those genes and proteins’ expression that were implicated in making a significant influence on the coagulation system, cholesterol biosynthesis, antimicrobial response plus a substantial impact on the xenobiotic metabolism signaling (Razali et al., 2015). The effect of “TSE,” tamarind seed coat extract in contrast to the toxicity of fluoride, by making use of the epithelial cells A549 of the lung, prevented the alterations induced by fluoride in the excess of (Ca(2+))I, generation of ROS, peroxidation of lipid, protein, and carbonyl content plus the antioxidant (superoxide dismutase, glutathione, glutathione peroxidase, catalase, and nitric oxide) parameters. It modulated activated change in the permeability transition pore opening, potential of mitochondrial membrane and in the release of Bax/Bcl‐2 ratio, cytochrome‐C, PARP‐1, and caspase‐3 expressions (Ameeramja et al., 2016).

Tamarind seed extract via restraining TRAP and MMP’s, exoglycosidases, cathepsins, and HAase, elevated activities exhibited the bone and cartilage protecting characteristic nature. Tamarind seed coat extract also moderated the augmented levels of the interleukins like (IL‐6 and L‐23), tumor necrosis factor, and also cyclooxygenase‐2 and interleukin (IL)‐1β, which are the inflammatory mediators. In addition to this, the administration of TSE alleviated the levels of and hydroperoxides and ROS, and maintained the endogenous antioxidant homeostasis via balancing the altered levels of the endogenous antioxidant markers (Sundaram et al., 2015). The leaf fluid extract of tamarind (TFE) on the blood cells of human at the dose of 40 mg/ml prevented the red blood cell membrane from the deleterious effects caused by the potential action of hydrogen peroxide (H_2_O_2_) (Gunaseelan, 2016). The alcoholic extract from tamarind seed coat prevented the irradiation of human fibroblast cells and protected them from damage. It also resulted in the cell cycle arrest and suppression of the secretion of matrix metalloprotein 1 and increased the glutathione concentration. This report thus concluded that tamarind seed coat extract is a potent antioxidant and can further prevent the skin fibroblast cells from the damage induced by UVA radiation (Phetdee, Rakchai, Rattanamanee, Teaktong, & Viyoch, 2014).

Another study was conducted on inflammatory bowel disease (IBD) in which acute colitis was induced by administration of dextran sulfate sodium at percentage level of 3% in the water of mice, for a period of 7 days. A compound named luteolin at doses 20 and 50 mg/kg of body weight significantly decreased the colon shortening and tissue damage that was demonstrated in histopathological evaluation. It also successfully reduced the inflammatory mediators’ expression, like IL‐6, iNOS, and TNF‐α. Colonic content of MDA also decreased significantly. In addition to this, activities of SOD and CAT as well as levels of Nrf2 and its several downstream targets including, HO‐1 and NQO1, were raised (Li, Shen, & Luo, 2016). Reactive sugar‐derived end‐product methylglyoxal abbreviated as MG put forth harmful effects by way of induction of oxidative stress. It then exaggerates a succession of diabetic impediments. An investigation reported that luteolin prevented MG prompted cell death and making of different factors, tumor necrosis factor, reactive oxygen species, cardiolipin peroxidation, and mitochondrial superoxide. It was found luteolin augmented the levels of the antioxidant enzyme Nrf**2** plus glutathione and diminished inhibition of the enzyme; heme oxygenase‐1. This revealed that pretreatment with luteolin reduced mitochondrial dysfunction and increased the (PPARs) peroxisome proliferator‐activated receptor **γ** coactivator 1α and nitric oxide levels, proposing that luteolin may bring mitochondrial biogenesis (Abbasi, Khosravi, Aidy, & Shafiei, 2016; Suh, Chon, & Choi, 2016).

Different antiepileptic drugs are known to delay the cognitive function, and for this reason, there is a vital need for such AEDs which do not have such consequence. The anti‐inflammatory and cytoprotective properties of flavonoid “luteolin” have been described by numerous studies but still no one has inspected the antiseizure potential of this compound. Induction of seizures was done by the daily injection of PTZ in rats, for a 36‐day period. The pretreatment of the other two groups was done with luteolin, at doses of 50 or 100 mg kg^−1^ day^−1^ given orally for 30 min prior to the chemical administration. For checking the effects, the seizure severity was scored and Morris water maze was used to evaluate cognitive function. Some other parameters studied were neuronal damage, oxidative stress, brain‐derived neurotrophic factor expression, and the phosphor‐activation pathway of the kinase. A protein plus the response element binding protein pathway of cyclic AMP was also measured in hippocampus of the rats. LU pretreatment suppressed the seizure induction, its duration and its severity following chemical injection. Furthermore, it reversed the cognitive damage, condensed the oxidative and neuronal damage, and amplified the phosphoactivation of CREB, PKA, and the expression of the brain‐derived neurotrophic factor (BDNF). The results obtained indicated that LU as a treatment, modality for epilepsy plus its consequences should be studied further (Zhen et al., 2016).

### 3.4 Antidiabetic

Several phytochemicals extracted from *Tamarindus* *indica* like alkaloids, flavonoids, saponins, glycosides, cardiac glycosides, triterpenes, and tannins expressively dropped raised blood glucose, among diabetic rats (Yerima, Anuka, Salawu, & Abdu‐Aguye, 2014). The *T. indica* polyphenol administration at doses of 120 and 240 mg/kg in male diabetic rats which were induced with STZ (streptozotocin) displayed the anti‐inflammatory action on NO and TNF‐α. Moreover, its administration on neogenesis of β‐cell gave promising effects and the concentration of mRNA’s SREBP‐1c was improved (Sole, Srinivasan, & Akarte, 2013). The flavonoids extracted from aqueous seed of tamarind showed insulin mimetic effect and hence increased glucose uptake. This happened as result of improved transporter genes of glucose which involved expression of GLUT gene family and certain factors involved in regulation including element involve in sterol regulation inducing SREBP proteins and in rat's liver mRNA 1c. The tamarind flavonoid administration lowered the TNF‐α upon enhancing the NO level of serum due to the glycated stage of hemoglobin. The antidiabetic effect of TSE on STZ‐induced diabetes resulted from a plethora of complex mechanisms comprising of β‐cell neogenesis, calcium handling, SREBP‐1c, and GLUT‐2, GLUT‐4 increased expression (Sole et al., 2013). Similarly, another investigation was carried to understand the effect of *Tamarindus* *indica* pulp aqueous extract (TIE) in diet‐induced obese Sprague‐Dawley rats. It was done at extract concentrations of 5, 25, and 50 in different groups of rats for 10 weeks after the implication of diet rich in fats showed obesity. The extract promisingly decreased the triglyceride and plasma cholesterol levels, LDL which was lipoprotein in low‐density, and HDL which was lipoprotein of higher density increased, along with weight of the body being reduced in rats. Levels of fatty acid synthase (FAS) enzyme and plasma leptin action were reduced, and the efficiency of the defense system of antioxidant increased momentously. The study depicted antiobesity results, as signposted by means of a noteworthy decrease in weights of adipose tissue, along with lowered degree of hepatic steatosis. The extract of tamarind has been proposed to be hepatoprotective, since it overturned the elevation level of plasma liver enzymes. It was thus accomplished that TIE amended the parameters that were related to obesity in the blood, liver, and adipose tissues in a rat model, most probably by modifiable metabolism of lipid and decreasing of levels of leptin and FAS plasma. Another experiment demonstrated TIE controlled dose effects, and 50 mg/kg dose showed protuberant end product and pursued with 25 mg/kg dose and thus 5 mg/kg (Azman et al., 2012).

Supplementation with tender tamarind leaves suggestively upgraded the profiles of lipids and carbohydrates, which were evident through the analysis of glucose and lipid plasma reduction, rates of peroxidation of lipid, improved content of hepatic glycogen, concurrent enhancement in the profiles of renal and hepatic tissue antioxidant profiles and hexokinase activity, and last but not least cholesterol excretion (Vasant & Narasimhacharya, 2012). *Tamarindus indica* seed aqueous extract was evaluated to be of nutraceutical worth at the dose estimated per day of the body weight of 20 mg per 0.5 ml distilled water per 100 g and was shown prevented results in insulin serum at fasting increment as well as levels of lipid profile markers TG, TC, VLDL, and LDL. HDL levels and fasting serum DHEAS decrease were prevented by its administration in experimental models (Shahraki, Harati, & Shahraki, 2011). Similarly, an investigation revealed that *Tamarindus* *indica* fruit pulp extract at dosage of 5% treatment used for hypercholestrolemic hamsters caused a decrease in the levels of serum total cholesterol by 50%, non‐HDL cholesterol by 73%, and triglyceride contents by 60%, and an increase in high‐density lipoprotein levels by 61% was achieved with treatment of extract. In vitro experiment demonstrated that the extract showed free radical ameliorating ability, as judged by the 2–2‐diphenyl‐1‐picrylhydrazyl (DPPH) and assays of radical superoxide and caused dwindled lipid peroxidation in serum (Martinello et al., 2006).

Similarly, in vitro exposure of peritoneal macrophages to a dose ranging from 0.2 to 200 μm/ml of *Tamarindus* *indica* extract expressively lessened to about 67% of nitric oxide production that was inducted in a concentration‐dependent manner by way of lipopolysaccharide as well as interferon gamma. Furthermore, the administration of plant's extract at 100–500 mg/kg to mice inhibited LPS, IFN gamma, and TPA prompted creation of separated peritoneal macrophages’ nitric oxide levels with no significant effect on weight of animals. Preliminary safety studies showed decrement in body weight only at the highest tested dose of 1,000 mg/kg but no fluctuations were found in hematological evaluations, weights of selected organs, and natural killer cell activity and serum chemistry. A noteworthy reduction in body weight was observed in mice that were given the doses of extract at 250 mg/kg or higher. Oral exposure to extract played no role in controlling formation of T‐cell‐regulated sensitization to HCA, and it was assessed by the dermal irritation to an acid (nonanoic acid) or lymphrried node assay (Hamidreza, Heidari, Shahraki, & Moudi, 2010; Komutarin et al., 2004). In a study carried out in streptozotocin‐induced diabetic rats, it was proposed that the aqueous extract of seed of *Tamarindus* *indica* expressively caused diminution in hyperglycemia as demonstrated by decreased blood sugar, glycogen levels, and glucose‐6‐phosphatase enzyme activity in addition with continuous monitoring of serum insulin levels (Maiti, Das, & Ghosh, 2005).

It was further reported that *Tamarindus* *indica* supplementation at the dose level of 80 mg per 0.5 ml water per 100 g body weight in diabetic rats resulted in worth‐mentioning reduction of blood sugar (fasting) levels after a period of 7 days. It was also demonstrated that continuous supplementation for a number of 14 days did not cause any noteworthy alteration in the factor as compared to control level. Momentous rise in liver and skeletal muscle glycogen content and the activity of liver enzyme glucose‐6‐phosphate dehydrogenase as compared to diabetic group were reported. Activities of some other enzymes comprising of hepatic enzyme glucose‐6‐phosphatase, hepatic, and renal glutamate pyruvate transaminase and glutamate oxaloacetate transaminase (GOT) were declined considerably in the group supplemented group as compared to the diabetic control group (Maiti et al., 2005).

Another evaluation reported that trypsin inhibitor extracted from tamarindus caused reduction in consumption of food and thus reduced weight gain. There was no difference in vivo true digestibility between control group and the other groups that were treated with the tamarindus trypsin inhibitor. It caused no significant alterations in the biochemical parameters regarding liver, pancreas, stomach, and intestine histology. The trypsin inhibitor group rats showed suggestively raised cholecystokinin hormone levels in contrast to animals that were given casein or water only (Ribeiro et al., 2015).

Nonalcoholic fatty liver disease is considered as series of pathological conditions characterized by fatty infiltration. It ranges from simple steatosis through nonalcoholic steatohepatitis to advanced stages of fibrosis and cirrhosis that result in the absence of alcohol consumption, any viral infection, or different other specific etiologies (Tan et al., 2013). As its strong association with obesity, type 2 diabetes mellitus, reduced glucose tolerance, arterial hypertension, and hypertriglyceridemia has been researched so far, NAFLD is thus universally considered as the hepatic demonstration of the deadly metabolic syndrome status these days. Insulin resistance is considered as the key pathophysiological hallmark for the metabolic syndrome (Yilmaz, 2012).

Another evaluation was done in the same context to evaluate prophylactic effect of the seed coat extract of the plant *Tamarindus* *indica*, on NAFLD (nonalcoholic fatty liver disease) induced by high‐fat diet following the administration on daily basis of the seed coat extract at doses of 45, 90, and 180 mg/kg body weight for a total period of approximately 6 weeks, induced in rats greatly assuaged the pathological alterations that were associated with the high‐fat diet‐induced nonalcoholic fatty liver disease (NAFLD) known as “hepatomegaly” raised the hepatic (liver) lipid and lipid peroxide levels, free fatty acids, and serum alanine aminotransferase levels plus the micro‐ and macrohepatic steatosis. It was observed that extract attenuated the pathologically disturbed manifested markers associated with high‐fat consumption. These evaluated parameters included raised hepatic lipid peroxides, fatty acid levels, micro‐ or macrohepatic steatosis, and serum alanine aminotransferase levels. It was observed that the treatment noticeably reduced the adiposity in tissues and body weight, and brought about improvement in the resistance of insulin and various other parameters (Sasidharan et al., 2014).

Another evaluation reported that obesity induced by cafeteria diet and antipsychotic drug was promisingly reduced by ethanolic extract doses of (50 and 100 mg/kg p.o.) for *Tamarindus* *indica*. The parameters that were diminished included the body weight, glucose levels, serum total cholesterol, and triglycerides. The decreased levels of HDL cholesterol were enhanced to a noteworthy level (Jindal, Dhingra, Sharma, Parle, & Harna, 2011).

Furthermore, the hypercholesterolemic hamsters showed a significant drop in the serum triglyceride, LDL and total cholesterol levels as a result of the administration of *Tamarindus* *indica* fruit pulp, whereas on the HDL levels among the treated rats, no significant effect was made. The lowering effect on lipid levels went together with a substantial upsurge in manifestation of the genes including Apo A1, LDL, and Abcg5 receptor and important diminution in the expression of a reductase namely, HMG‐CoA reductase and levels of MTP genes. Hypocholesterolemic effect was shown by increase in the cholesterol efflux, enhanced the uptake and clearance of LDL, and hence, caused suppressed triglyceride accumulation and inhibition of cholesterol biosynthesis in rats (Lim et al., 2013). It also caused reduced enzyme GPx activity and bilirubin content in feces of rats, and increased red blood cell parameters in heat‐stressed broilers (Aengwanich & Suttajit, 2010).

### 3.5 Cardiovascular role

*Tamarindus* *indica* fruit is rich in flavonoids and polyphenols. It moderately shows the antioxidant effects also. The epidemiological studies now have also revealed the fact that the intake of flavonoids from fruit as well as vegetable sources has an immensely worth‐mentioning effect on the cardiovascular health of human beings (Lim et al., 2013). The fruit of *Tamarindus* *indica* shows antioxidative and hypocholesterolemic properties by increasing, in liver, the expression of Apo‐A1, LDL, and ABCG5 receptor genes and by the inhibition of the MTP gene expression. It enhances the excretion of cholesterol and decreases its biosynthesis and also from the peripheral tissues, increases the intake of LDL‐cholesterol, and thus prevents the triglycerides accumulation in the liver. It also prevents the damage caused by oxidation, which is the main risk factor of atherosclerosis, to LDL‐cholesterol. It was indicated by Martinello et al. (2006 that the fruit extract of T. indica decreased 50% of the serum total cholesterol, 73% of LDL, and 60% of triglyceride and improved the percentage of HDL (61%). It prevents aortic atherosclerosis in high‐cholesterol diet group by the activation of antioxidant defense mechanism (Martinello et al., 2006). The seed of T. indica through its polyphenol, flavonoid, anthocyanin, tannin, and oligomeric proanthocyanidin displays the antioxidant effect. The immunomodulatory effect was shown by the polysaccharides that were isolated from the seed of T. indica through increasing the process of phagocytosis, decreasing the proliferation of cells, and by inhibiting the migration of leukocytes (Chong, Abdul‐Rahman, Abdul‐Aziz, Hashim, & Junit, 2012). The effect, by which triglycerides started decreasing, is associated with the extract's epicatechin content. This compound increases the neutral and acidic sterols; the total fatty acids excreted through the faces, and it thus shows hypolipidemic effect. Therefore, as a nutritional support in the patients with high levels of blood cholesterol, the seeds and fruit of tamarind are highly suggested (Landi Librandi et al., 2007).

IPRT also known as isoproterenol (1‐(3,4‐dihydroxyphenyl)‐2‐isopropylaminoethanol hydrochloride) is a synthetic catecholamine and a β‐adrenergic agonist that has been established to produce extreme stress in the myocardium leading to myocardial infarction, and it leads to myocardial necrosis which roots to cardiac dysfunction, increased lipid peroxidation besides an elevated level of myocardial lipids and altered activities of the cardiac enzymes and antioxidants, when administered in supramaximal doses (Karthikeyan, Bai, & Devaraj, 2007).

T. indica fruit pulp extract was found to be responsible to bring about decrease in profusion of proteins which were taking part in the polyamines and nucleic acid's metabolism of liver HepG2 cells. These have not been formerly reported, and also their rationale is not fully understood, as far as we have knowledge about it.

Conversely, the decreased load of the ethanolamine phosphate cytidylyltransferase commonly referred to as PCYT2 enzyme that is rate‐limiting, which in the biosynthesis of phosphoethanolamine, catalyzes the conversion of phosphoethanolamine to cytidylyl phosphoethanolamine in HepG2 cells that were exposed to the extract of tamarind fruit, may perhaps concede the ease of use of phospholipid which for prostaglandins’ production, stores the arachidonic acid. This therefore can probably explain the *Tamarindus indica*'*s* anti‐inflammatory action that was also previously reported (Rimbau, Cerdan, Vila, & Iglesias, 1999).

### 3.6 Anti‐inflammatory activity

Inflammation is a typical protective response of the body toward tissue injury that is caused by physical trauma, noxious chemicals, or by microbiological agents. It is actually the body's effort to inactivate or destroy the invading organisms, removes the irritants, and sets the stage for the repair of tissues (Khan, Noorulla, Muqtader, Roshan, & Sadath, 2013). Synthetic drugs that are commonly used for the treatment of pain and inflammation like nonsteroidal anti‐inflammatory drugs and corticosteroids provide symptomatic and ephemeral relief. In addition, their long‐term uses are associated with several serious and undesirable effects. Hence, the discovery of new and safe analgesic and anti‐inflammatory drug is indispensable. The healing power of tamarind was first mentioned in the traditional Sanskrit literatures (Khan et al., 2013).

Luteolin, a phytochemical that is actually a flavonoid, is acknowledged as an important inflammation curbing compound of the plant *Artemisia* *asiatica*. Several reports have enlightened the ability of luteolin regarding the suppression of inflammation in a number of circumstances associated with inflammation. Nevertheless, the exact mechanism has not been figured out yet. In this study, the anti‐inflammatory way of action of luteolin in the different potential macrophages from *A. asiatica* was inspected by making use of a luciferase reporter gene assay, immunoblotting analysis, and enzyme assays. Luteolin administration depressed the secretion of a compound named nitric oxide and prostaglandin in a dose‐dependent manner; further it decreased the intensities of transcripts of mRNA related to inducible nitric oxide synthase, cyclooxygenase‐2, and tumor necrosis factor. Luteolin demonstrated a significant nitric oxide ameliorative activity and further suppressed the translocation of nuclear factor‐kappa b (p50 and p65) by way of Src and Syk cordon but no effect was shown on other nitrogen‐related activated kinases. The overexpression of wild‐type Src and point mutants thereof and the molecular modeling studies proposed that the luteolin‐binding site in Src may be considered luteolin‐building pocket. These results strongly suggest that by culminating this nuclear factor signaling by way of blocking the ATP binding in and Syk and Src, the compound luteolin may exert its anti‐inflammatory action (Lee, Jeong, Kim, & Cho, 2015).

Procyanidin B2‐mediated inhibition of inflammasome activation includes the NF‐κB signaling pathway inactivation, the first stage required for the transcription of inflammasome precursors, due to the inhibition of p65 nuclear expression and DNA binding, resulting in the transcriptional repression of the target genes, such as COX_2_, **i**NOS, and production of IL‐6 and NO. Moreover, procyanidin B2 decreases NLRP3 and pro‐IL‐1β cytoplasmic pools, limiting the components of inflammasome activation and impeding the inflammasome assembly and caspase‐1 activation, and secretion of active IL‐1β at the end. Procyanidin B2, during LPS‐induced acute inflammation in human macrophages, inhibits the activation of inflammasome and IL‐1β secretion (Martinez‐Micaelo, González‐Abuín, Pinent, Ardévol, & Blay, 2015).

## 4 MISCELLANEOUS PROPERTIES

In the traditional herbal Indian medicine system, several plants have been employed extensively as a treatment for snake bites. In another investigation that depicted the potentiality of *Tamarindus* *indica* seed extract on the enzymatic and pharmacological propensity induced by venom of *V. russelli,* the extract of tamarind seed inhibited the protease, amino acid oxidase hyaluronidase, PLA (2), and 5'‐nucleotidase enzymatic activities of the venom in a manner that was dose dependent. These are majorly the hydrolytic enzymes that are considered responsible for the initial and important effects on envenomation such as inflammation, hypotension, and local tissue damage. Additionally, the extract acted to neutralize the breakdown of the human fibrinogen beta chain and hemolysis that occurred indirectly by venom. It was further revealed that the seed extract showed a moderate response regarding the clotting time and prolonged it only to a small extent. Hemorrhage, edema, and myotoxic effects including necrosis that was induced by the venom were neutralized considerably when several doses of the extract were preincubated with the venom before the analysis (Ushanandini et al., 2006). Alternatively, those animals which were given the extract, 10 min after injecting the venom, were protected from the toxicity induced by the venom. As the extract inhibits the activity of enzymes for hydrolysis and pharmacological aspects, so it can perhaps be employed as a rich source of potential inhibitors of phospholipases A2 PLA(2), hyaluronidases, metalloproteinases plus serine proteases, and 5‐nucleotidases, the enzymes involved in numerous physiopathological diseases of the humans and animals and as an effective alternative treatment to serum therapy (Parvez et al., 2003).

Arthritis is characterized by the degradation of articular cartilage and subchondral bone, which is accompanied by inflammation, pain, and immobility. Articular cartilage, containing chondrocytes, is a specialized form of connective tissue that is encased by components of the extracellular matrix (ECM) which include most importantly collagen, proteoglycans, aggrecans, and hyaluronic acid. The Arthritis’ pathogenesis entails the most important articular cartilage enzyme degradation, like matrix metalloproteinases, aggrecanases, and hyaluronidase and exoglucosidases. Moreover, different reactive oxygen and nitrogen species as well as several proinflammatory mediators including interleukin (IL)‐1β, IL‐23, cyclooxygenase 2, and tumor necrosis factor‐α that act as cytokines play important role by way of triggering very potent signaling cascades for inflammation (Campo et al., 2012; Hemshekhar et al., 2012).

In another investigation, it was proposed that the oral administration of tamarind extract efficiently abridged the swelling of paw. Furthermore, it also protected bone and cartilage deterioration by assuaging increased levels of the different degrading enzymes of cartilage including metalloproteinases in addition to many others. The bone‐resorbing enzymes of different types just like cathepsins, exoglycosidases, ALP, and ACP, these enzymes for the most part, are proven significant in reducing the collagen and hyaluronic acid likewise, which are the backbones of articular cartilage. Numerous studies conducted previously have explained in arthritic patients, the amplified activities of these bone‐resorbing enzymes in the blood serum and synovial fluid (Wu et al., 2011). The proinflammatory mediators and ROS have been recognized as extremely menacing, chief nonenzymatic factors that are responsible for the Arthritis’ progression. They also make it even worse, by provoking the immunological cell signal transmission cascade. In addition, cytokines like IL‐1β and TNF‐α are also acknowledged as the two most effective mesenchymal cells’ stimulators, such as osteoclasts, chondrocytes, and synovial fibroblasts, which discharge such matrix metalloproteinases MMP’s that damage the tissues (Lee et al., 2015; Yoon et al., 2013).

Consequently, the aforementioned events encourage the osteoclasts toward releasing the bone‐resorbing enzymes such as phosphatase, phosphatases, and cathepsins, which are also tartrate resistant. Hyaluronic acid oligosaccharides, numerous peptides, and its derivative end products and collagen that are recognized as being proinflammatory are verified to deteriorate the malady. Stress, which is produced as result of oxidation during arthritis, has also been proposed to impart a gradual influence on the components of blood and on organs of vital functions. Therefore, the prevention of cartilage and bone disintegration, acute/chronic inflammation, and oxidative stress is of extreme importance in order to promote the pathogenesis of arthritis (Campo et al., 2012; Kundu et al., 2012). A study was conducted in order to determine the arthritis curbing worth of seed extract of tamarind and displayed the protective nature of cartilage and bone by way of hindering the raised potential actions of metalloproteinases, cathepsins, and exoglycosidases. In addition, it was also observed that extract lessened the amplified levels of mediators like interleukin (IL), namely 1β, 6, 23, cyclooxygenase‐2, and tumor necrosis factor‐α (TNF‐alpha). It also decreased augmented levels of oxygen species most importantly hydroperoxides, hence, preserved the body's antioxidant levels by augmenting the increased levels of various endogenous biomarkers of antioxidants (Sundaram et al., 2015).

## 5 CONCLUSIONS

*Tamarindus indica* in addition to its antioxidant effect also possesses the blood glucose‐lowering effect, a significant protective effect on renal complications that are associated with hyperglycemia and boosts the immune system as well. This shows that tamarind has a strong ability to decrease the oxidative stress and related disturbances plus it is useful against a number potential health risking disorders which include cancer, cardiovascular diseases, arthritis, diabetes, epilepsy, nonalcoholic fatty liver disease, and inflammatory bowel disease. The following review summarizes the literature in an explicit way relating to tamarind and its possible allied health claims.

## CONFLICT OF INTEREST

The authors declare no conflict of interest.

## ETHICAL APPROVAL

This study has nothing to do with human and animal testing.
